The article "Aldehyde Dehydrogenase 2 (ALDH2) Elicits Protection against Pulmonary Hypertension via Inhibition of ERK1/2-Mediated Autophagy" was published in 2022. Journal: Oxid Med Cell Longev.

# Aldehyde Dehydrogenase 2 (ALDH2) Elicits Protection against Pulmonary Hypertension via Inhibition of ERK1/2-Mediated Autophagy

**DOI:** 10.1155/2022/2555476

**Published:** 2022-06-20

**Authors:** Suchi Chang, Jian Wu, Jifu Jin, Huairui Shi, Rifeng Gao, Xiao Li, Daile Jia, Xiaolei Sun, Tiantong Ou, Ji'e Yang, Aijun Sun, Junbo Ge

**Affiliations:** ^1^Department of Cardiology, Zhongshan Hospital, Fudan University, Shanghai Institute of Cardiovascular Diseases, Shanghai 200032, China; ^2^Key Laboratory of Viral Heart Diseases, Chinese Academy of Medical Sciences, National Health Commission, Shanghai 200032, China; ^3^Institutes of Biomedical Sciences, Fudan University, Shanghai 200032, China; ^4^Department of Cardiology, Shanghai East Hospital, School of Medicine, Tongji University, Shanghai 200092, China

## Abstract

Pulmonary hypertension (PH) is caused by chronic hypoxia that induces the migration and proliferation of pulmonary arterial smooth muscle cells (PASMCs), eventually resulting in right heart failure. PH has been related to aberrant autophagy; however, the hidden mechanisms are still unclear. Approximately 40% East Asians, equivalent to 8% of the universal population, carry a mutation in Aldehyde dehydrogenase 2 (ALDH2), which leads to the aggregation of noxious reactive aldehydes and increases the propensity of several diseases. Therefore, we explored the potential aspect of ALDH2 in autophagy associated with PH. *In vitro* mechanistic studies were conducted in human PASMCs (HPASMCs) after lentiviral ALDH2 knockdown and treatment with platelet-derived growth factor-BB (PDGF-BB). PH was induced in wild-type (WT) and ALDH2-knockout (ALDH2^−/−^) mice using vascular endothelial growth factor receptor inhibitor SU5416 under hypoxic conditions (HySU). Right ventricular function was assessed using echocardiography and invasive hemodynamic monitoring. Histological and immunohistochemical analyses were performed to evaluate pulmonary vascular remodeling. EdU, transwell, and wound healing assays were used to evaluate HPASMC migration and proliferation, and electron microscopy and immunohistochemical and immunoblot assays were performed to assess autophagy. The findings demonstrated that ALDH2 deficiency exacerbated right ventricular pressure, hypertrophy, fibrosis, and right heart failure resulting from HySU-induced PH. ALDH2^−/−^ mice exhibited increased pulmonary artery muscularization and 4-hydroxynonenal (4-HNE) levels in lung tissues. ALDH2 knockdown increased PDGF-BB-induced PASMC migration and proliferation and 4-HNE accumulation *in vitro*. Additionally, ALDH2 deficiency increased the number of autophagosomes and autophagic lysosomes together with autophagic flux and ERK1/2-Beclin-1 activity in lung tissues and PASMCs, indicating enhanced autophagy. In conclusion, the study shows that ALDH2 has a protective role against the migration and proliferation of PASMCs and PH, possibly by regulating autophagy through the ERK1/2-Beclin-1 pathway.

## 1. Introduction

Pulmonary hypertension (PH) is a serious, progressing syndrome that contributes to enhanced pulmonary vascular resistance, dyspnea, right-sided heart failure, and ultimately the loss of life [1, 2]. Although several medications have lately been shown to have some favorable therapeutic effects on PH [3], none have shown sufficient efficacy [4]. PH is commonly induced by chronic hypoxia and is frequently observed in various chronic lung diseases and metabolic dysfunction [5], such as chronic obstructive pulmonary disease, high-altitude pulmonary vascular disease, and obstructive sleep apnea syndrome [6]. Pulmonary vascular remodeling is central to the pathobiology of PH. It is principally characterized by medial thickening and increased muscularization of the pulmonary arteries due to enhanced migration and proliferation of pulmonary artery smooth muscle cells (PASMCs) [7, 8]. Likewise, excessive migration and proliferation of PASMCs are the hallmark features of pulmonary vascular remodeling [9]. Therefore, it is critical to identify the underlying pathological mechanisms of PASMCs to prevent and treat of PH.

Aldehyde dehydrogenase 2 (ALDH2) is a mitochondrial isoform of the ALDH superfamily that includes 19 subtypes [10]. This metabolic enzyme plays essential roles in the oxidation and detoxification of reactive aldehydes, including the ethanol metabolites acetaldehyde and 4-hydroxynonenal (4-HNE), in various organs and cells [11]. It is well documented that ALDH2 protects against myocardial damage by clearing toxic aldehydes generated from 4-HNE [12]. Our previous studies have demonstrated its fundamental role in cardiovascular circumstances, such as heart failure, myocardial infarction, pressure overload, and ischemia/reperfusion injury [13–16]. However, ~40% of the East Asian population (equivalent to ~8% of the universal population) carry a mutation of ALDH2, which leads to the defective enzyme activity of ALDH2 and consequently increases the propensity of several diseases [17]. Recently, it has been shown that ALDH2 deficiency is involved in PASMC proliferation associated with PH [18, 19]. However, whether it elicits protective effects against PH and right ventricular remodeling remains to be elucidated in addition to the underlying signaling mechanisms.

Autophagy is a lysosome-dependent cellular program for the degradation and turnover of impaired cytoplasmic substrates via a self-degradation pathway [20]. Autophagy functions as a fundamental process in sustaining cellular homeostasis, and its dysregulation is associated with various cardiopulmonary diseases, including load-induced cardiac remodeling, ischemic cardiac remodeling, chronic obstructive pulmonary disease, and PH [21]. Nevertheless, the argument remains whether autophagy serves as a protecting or worsening process because both excessive and insufficient autophagy contributes to cell death [22, 23]. Although some studies have reported that autophagy inhibition via deletion of the autophagic protein LC3B enhances hypoxia-induced PASMC proliferation [24], other studies have found that its pharmacological inhibition suppresses PASMC proliferation [25]. Moreover, the molecular network underlying autophagy is intrinsic and is linked to different unique signaling pathways; thus, its fine modulation may profoundly impact the pathogenesis of certain diseases. In particular, the PI3K-AKT-mTOR and ERK1/2-Beclin-1 signaling pathways have been shown to modulate autophagy under specific conditions [25, 26]. Nevertheless, the function of autophagy in PH is not been thoroughly recognized so far, and the involvement of ALDH2 remains unclear. Therefore, the present study examines the abnormal migration and proliferation of PASMCs associated with ALDH2 deficiency while focusing on autophagy in PH.

## 2. Materials and Methods

### 2.1. Animal Models

Male C57BL/6 mice, eight weeks of age with a weight of 20–22 g, purchased from the Shanghai Jiesijie Laboratory Animal Centre (Shanghai, China), and paired ALDH2 knockout (KO) male mice developed as reported [27], were used in our study. Genotypes of the mice were identified using western blotting. Mice were exposed to vascular endothelial growth factor receptor inhibitor, SU5416, and under hypoxic conditions for three weeks to induce pulmonary artery hypertension and were maintained on a 12/12 h dark/light cycle with ad libitum access to water and diet. All animal experiments were authorized by the University Committee on the Care and Use of Laboratory Animals and were performed according to the guidelines of the Animal Ethics Committee of Fudan University.

### 2.2. Echocardiography

Transthoracic echocardiography was demonstrated on the mice after three weeks of HySU, utilizing a Vevo 2100 (VisualSonics, Toronto, Canada) supplied with a 30 MHz transducer. Mice were settled on a warming pad and anesthetized with 2% isoflurane. Right ventricular ejection fraction (RVEF), pulmonary artery acceleration time (PAT), and PAT/pulmonary ejection time (PET) were then acquired.

### 2.3. Right Ventricular Pressure Measurement

After echocardiography, the right ventricular systolic pressure (RVSP), equivalent to the pulmonary arterial pressure, was measured. Briefly, under 2% isoflurane, a longitudinal skin incision was made. After tissue separation, the right external jugular vein was unveiled to insert a Millar micromanometer (1.4F, type SPR 835; Millar Instruments, Houston, TX type). Once the catheter arrived at the right ventricle, the right ventricular pressure was recorded using a Power-Lab system (AD Instruments, Castle Hill, NSW, Australia).

### 2.4. Histological Examination

After catheterization, the mice were euthanized by cervical vertebral luxation under deep anesthesia. Hearts and lungs were harvested for further examination. RV hypertrophy was defined as the ratio of the weight of the RV free wall to the weight of the left ventricle plus septum.

### 2.5. Electron Microscopy

Mouse heart and lung tissues (≤1 mm^3^) were fixed with 2.5% PIPES-buffered formaldehyde glutaraldehyde immediately after dissection. Following fixation with 1% osmium tetroxide, graded alcohols were used for the dehydration of heart and lung tissues. After fixing in Epon Araldite, tissues were prepared and stained with 3% uranyl acetate and lead citrate. CM-120 transmission electron microscope (Philips, Netherlands) was used to examine the results.

### 2.6. Histological Staining and Immunohistochemistry

Formalin-fixed tissues were fixed with paraffin and cut (3–5 *μ*m thickness) on a microtome for hematoxylin and eosin (H&E, histological measurement), wheat germ agglutinin (WGA, for cardiomyocyte size), and Masson's trichrome (for fibrosis) staining. Vascular muscularization percentage, right ventricular cardiomyocyte cross-sectional area, and fibrosis area were measured accordingly. For immunofluorescence staining, after incubating sectioned tissues with the primary antibodies (4-HNE and LC3) at 4°C overnight, they were washed three times and then incubated with a secondary antibody at 20–24°C for 1 h. Finally, the nuclei were counterstained using 4′,6-diamidino-2-phenylindole (DAPI, Beyotime Biotechnology, China). The stained sections were analyzed and recorded using an optical microscope (FSX-100; Olympus, Tokyo, Japan) and a fluorescence microscope (Olympus, Japan). ImageJ 1.47v (U.S. National Institute of Health, Bethesda, MD, USA) was used to quantify the percentage of positive area.

### 2.7. Cell Culture

Human PASMCs were obtained from ScienCell Research Laboratories (Carlsbad, CA, USA) and cultivated at 37°C 5% CO_2_ atmosphere in smooth muscle cell medium (ScienCell, Carlsbad, CA, USA) supplied with 100 *μ*g/mL streptomycin, 100 U/mL penicillin, smooth muscle cell growth supplement (ScienCell, Carlsbad, CA, USA), and 5% fetal bovine serum. The cell medium was refreshed regularly, and cells were subcultured after achieving 70%–80% confluence. Cell numbers were determined using a hemocytometer.

ALDH2 knockdown cells were cultivated by transfection with lentivirus [28], and control cells were transfected with negative control lentivirus (NC). Successful depletion of ALDH2 was confirmed by western blotting. Since the regulation of platelet-derived growth factor- (PDGF-) BB fundamentally participates in the pathogenesis of PH [29, 30], and the elevated activity of PDGF results in excessive migration and proliferation of PASMC, as observed in human and previous experimental PAH models [31, 32], the *in vitro* model of PH [33] was developed by pretreatment with 20 ng/mL PDGF-BB (MedChemExpress, New Jersey, USA) for 24 h.

### 2.8. Scratch Assay

An *in vitro* scratch assay was performed to examine cell migration of HPASMCs. Photographs were taken before and after a “scratch” was created in a cell plate at a 24-hour interval. The migration rate of the cells was evaluated and quantified by the differences in cell migration to close the scratch.

### 2.9. Transwell Assay

Transwell assay was carried out in a 24-well transwell chamber (Corning Incorporated Life Sciences, MA, USA). ALDH2^−/−^ and control HPASMCs (1 × 10^5^ cells) were cultivated in the upper compartment in a serum-free medium. A complete medium with 0 or 20 ng/mL PDGF-BB was supplemented to the lower compartment. Migrated cells were stained with 0.1% crystal violet dye (Biyuntian, Shanghai, China) after incubation at 37°C environment for 24 hours, and images were captured for quantification.

### 2.10. Measurement of Cell DNA Synthesis

DNA synthesis, indicating cellular proliferation, was performed using the EdU kit (Beyotime, C0071S). After seeding in a 6-well plate for 24 h of serum deprivation, ALDH2^−/−^ and control HPASMCs were intervened with or without PDGF-BB (20 ng/mL) for 24 hours. The cells were stained with 50 *μ*mol/L 5-ethynyl-2′-deoxyuridine (EdU) and DAPI for observation using a fluorescence microscope (ZEISS Group).

### 2.11. Confocal Fluorescence Microscopy

ALDH2^−/−^ and control PASMCs were transfected with mRFP-GFP-LC3 adenoviral vectors (HanBio Technology, Shanghai, China) following the manufacturer's protocols. Due to the different pH stability of fluorescent proteins, the GFP fluorescent signal, but not the mRFP fluorescent signal, could be diminished in the acidic environment inside lysosomes. In merged images, red and yellow puncta represent autolysosomes and autophagosomes, respectively, and the increase in yellow and red puncta represents an increase in autophagic flux upon examination [34]. Afterward, experimental groups were intervened with PDGF-BB (20 ng/mL), as previously described [33]. After fixing with 4% paraformaldehyde, cells were blocked with glycerol, and LC3 localization was visualized using a confocal fluorescence microscope (Nikon TE2000, Tokyo, Japan).

### 2.12. Western Blot Analysis

Proteins of both mouse tissue and HPASMCs were extracted [35] and fractionated using 12% sodium dodecyl sulfate-polyacrylamide gel electrophoresis. After that, the proteins were transferred to polyvinylidene difluoride membrane (Millipore) and blocked with 5% bovine serum albumin. Next, the membranes were incubated with the following primary antibodies: *β*-actin (13000; Wei'ao), rabbit anti-mouse polyclonal antibody, anti-4-hydroxynonenal (Abcam, 11000), anti-ALDH2 (Abcam, 11000), anti-cyclin D1 (CST, 11000), anti-PCNA (CST, 11000), anti-LC3 (CST, 11000), anti-p62 (CST, 11000), anti-ATG5 (Abcam, 11000), anti-ATG7 (Abcam, 11000), anti-Beclin1 (CST, 11000), anti-pPI3K (CST, 11000), anti-PI3K (CST, 11000), anti-pAKT (CST, 11000), anti-AKT (CST, 11000), anti-pmTOR (CST, 11000), anti-mTOR (CST, 11000), and anti-ERK1/2 (CST, 11000). Afterward, the membranes were washed three times using phosphate-buffered saline with Tween-20, and the samples were incubated with anti-mouse or anti-rabbit secondary antibodies (Kangcheng, 13000). Finally, the blots were analyzed using a chemiluminescence detection system (Thermo Fisher Scientific) and quantified using ImageJ gel analysis software.

### 2.13. Statistical Analysis

All quantification analyses of the experiments were performed with GraphPad Prism 9.2.0. Experimental data are presented as the mean ± SEM for all analyses. One-way ANOVA or two-way ANOVA with Bonferroni correction was utilized for multiple group analysis. A *p* value of *p* < 0.05 was considered to be of statistical significance.

## 3. Results

### 3.1. ALDH2 Deficiency Exacerbates Right Ventricular Pressure and Dysfunction in PH

Considering RVSP was commonly used to estimate pulmonary arterial pressure, we first investigated whether ALDH2 was involved in the changes in RVSP after 3 weeks of HySu treatment. Wild-type (WT) mice in the PH group (WT PH) exhibited elevated RVSP in comparison to those in the control group (WT CON). The significant increase in RVSP was more pronounced in ALDH2-knockout (ALDH2^−/−^) mice of the PH group (KO PH) compared with WT mice of the PH group (WT PH) (Figure 1(a)). In consistency, the echocardiographic analysis showed that HySu treatment caused impairment of RVEF and decrement of PAT and PAT/PET (Figures 1(b)–1(e)), while the changes were further aggravated in the ALDH2^−/−^ mice, suggesting ALDH2 preserves right ventricular pressure and function in PH mice.

### 3.2. ALDH2 Deficiency Worsens the Extent of PH and Its Effects on Right Ventricular Remodeling and Cardiomyocytes

The elevation of RVSP induces right ventricular remodeling which could progress to right ventricular dysfunction. Therefore, we evaluated the morphological alterations in the cardiac tissues of the mice were investigated to better understand the effects on the heart due to the extent of PH. The gross appearances of the hearts, the mid transverse sections of the H&E stained hearts, and the right ventricular hypertrophy index all indicated that the RV hypertrophy of PH mice was more pronounced in comparison with that in the control mice, while the ALDH2^−/−^ PH mice exhibited the most significant elevation (Figures 2(a) and 2(b)).

We then explored whether similar changes can be found in the right ventricular cardiomyocytes from a microscopic perspective. WGA staining of the RV showed that the cross-sectional area of the cardiomyocytes in the PH group was larger than that in the control group, and the difference was even more significant in the ALDH2^−/−^ PH group (Figure 2(e)). Further assessment of the RV with transmission electron microscopy revealed that the control group exhibited regularly arranged muscle bundles and normal-sized cardiomyocytes with normal mitochondria. The WT PH group also exhibited regularly arranged muscle bundles, but the mitochondria were slightly swollen. In contrast, the KO PH group exhibited disrupted muscle bundle arrangement as well as evident mitochondrial edema (Figure 2(c)). Furthermore, cardiac fibrosis of RV showed congruent results, with the most prominent fibrosis revealed in the ALDH2^−/−^ PH group (Figure 2(d)).

### 3.3. ALDH2 Deficiency Exacerbates Pulmonary Vascular Remodeling and Oxidative Damage in PH

The remodeling of the pulmonary vessel is typically induced by PH. Although functioning as a compensated mechanism to counteract the elevated PH, pulmonary vascular remodeling produces increased vascular resistance and leads to RV dysfunction in the long term [7]. Therefore, the analysis of pulmonary vascular remodeling in lung tissue was performed. Consistent with hemodynamic findings, in PH mice, the structural analyses of pulmonary arterioles by H&E staining indicated the ratio of normal (without muscularization) blood vessels was strikingly decreased in both WT and ALDH2^−/−^ mice, while ALDH2 deficiency showed a more noteworthy decrease. In contrast, the percentages of fully muscularized vessels in both WT PH and KO PH mice were significantly higher than that in the control group, while ALDH2 deficiency further promoted muscularization. (Figure 3(a)). Correspondingly, pulmonary fibrosis expressed by trichrome staining and western blot analysis of alpha-smooth muscle actin (*α*-SMA) and fibronectin were both aggravated by the knockout of ALDH2 (Figures 3(b) and 3(c)). 4-HNE is a sensitive marker of oxidative damage [36], which is oxidized and detoxified by ALDH2. The 4-HNE immunohistochemical staining showed that the proportion of 4-HNE–positive cells in the lungs of the PH mice was higher in the lungs of the control group, while it was the highest in the ALDH2 deficient group (Figure 3(f)). Successful knockdown of ALDH2 was verified by western blot analysis (Figure 3(d)). Consistent *in vitro* results were obtained by western blot analysis in HPASMCs treated with PDGF-BB. Specifically, an obvious increment in the expression of 4-HNE was visualized (Figure 3(e)).

### 3.4. ALDH2 Knockdown Accentuates PASMC Migration and Proliferation in PH

The structural alterations within the remodeling of the pulmonary vessel are caused mainly by the migration and proliferation of PASMC [2]. Therefore, we investigated whether the effects of ALDH2 were underscored by changes in the migration and proliferation ability of PASMC. The wound-healing assay revealed that 24 h of PDGF-BB intervention, the migration ability of HPASMC was promoted with a reduced wound area, compared with that in the control group, and the difference was more conspicuous when ALDH2 was knocked out (Figure 4(a)). Subsequently, the transwell experiment revealed that, after PDGF-BB intervention, the number of migrating cells increased in comparison with that in the control group. Knockdown of ALDH2 further augmented the number of migrating cells (Figure 4(b)).

The effect of ALDH2 knockdown on the proliferation of PASMCs was also observed in two parts. First, the EdU assay demonstrated a higher fluorescence intensity in the Lenti-NC PDGF group than that in the control group, while the intensity in the ALDH2 knockdown HPASMC group was more significant (Figure 4(d)). Subsequent western blot assay after 24 h of PDGF-BB treatment demonstrated significantly elevated levels of proliferation-related proteins, proliferating cell nuclear antigen (PCNA), and cyclin D1 in PDGF-BB-treated groups than those in the control groups. Moreover, ALDH2 knockdown resulted in a more significant increase in these protein levels (Figure 4(c)). These findings indicated that ALDH2 knockdown enhanced PASMC proliferation.

### 3.5. ALDH2 Deficiency Alters Pulmonary Autophagy Levels in Response to PH

The aberrant autophagic response is important in the pathogenesis of PH development [37]. Therefore, we determined whether autophagy is involved in the underlying mechanisms of worsening PH after ALDH2 deficiency. Electron microscopy assessment revealed no abnormal changes in the lungs of WT CON and KO CON mice; however, autophagosomes appeared in the lungs of mice in the WT PH and KO PH groups, particularly in the ALDH2-deficient lungs (Figure 5(a)). The effects of ALDH2 knockout on the autophagic response in the lung tissue were also evaluated using immunohistochemistry. Significantly higher LC3B expression was detected in mice in the WT PH and KO PH groups compared with the mice in the control group, suggesting an increased level of autophagy in the lungs of these mice. However, this difference was substantially higher in the KO PH group in comparison with that in the WT PH group, proposing that ALDH2 acts as an important factor in the autophagy response in PH (Figure 5(b)).

Furthermore, the autophagic response of HPASMC was further examined using confocal fluorescence microscopy. HPASMC was transduced with autophagic LC3 double-labeled adenovirus to observe morphological and autophagic flux alterations in response to PDGF-BB treatment and ALDH2 knockdown. Consistent with the previous results, the cells became larger and wider after PDGF-BB treatment, and these effects were further enhanced by ALDH2 knockdown. Alterations in autophagic flux were observed by confocal microscopy, and the number of autophagosomes significantly increased after PDGF-BB treatment, especially in the cells with ALDH2 knockdown (Figure 5(c)). Additionally, the western blot analysis revealed increased expression of LC3B, ATG5, ATG7, and Beclin-1 after PDGF-BB intervention, especially after ALDH2 knockdown (Figure 5(d)).

### 3.6. ALDH2 Deficiency Stimulates the Autophagy-Inducing ERK1/2 Signaling Pathway in PH

Autophagy is a multifaceted biological metabolic progression, which is regulated by several distinct signaling pathways, with the mitogen-activated protein kinase ERK1/2 and the PI3K-AKT-mTOR signaling pathways considered most critical [38]. Here, we determined whether ERK-1/2 and PI3K-AKT-mTOR signaling pathways were responsible for the previously-stated findings on autophagic alterations. As anticipated, ERK1/2 was considerably upregulated by PDGF-BB intervention and was further stimulated by the knockdown of ALDH2 in the PASMC. However, while challenged with PDGF-BB, the PI3K-AKT-mTOR signaling pathway was not suppressed as expected (Figures 5(e) and 5(f)).

## 4. Discussion

Recent studies have indicated that autophagy is a primordial determinant of health, suggesting autophagy regulation as a favorable approach for the prevention or treatment of common phenotypic abnormalities in various human diseases [39]. Although ALDH2 has been shown to have essential roles in the development of cardiopulmonary disease in both experimental and clinical backgrounds [13–16, 40], little is known regarding its role in PH, right ventricular remodeling, and the underlying autophagy-dependent mechanisms. In this study, we demonstrated that ALDH2 deficiency exacerbates pulmonary artery muscularization, right ventricular hypertrophy, fibrosis, and right-sided heart failure by regulating autophagy. The adverse effects of ALDH2 deficiency include the overt accumulation of 4-HNE and the considerable exacerbation of PASMC migration and proliferation. Mechanistically, enhanced autophagy is involved in PASMC migration and proliferation, and ALDH2 deficiency further induces autophagic activity via increased ERK1/2 activity.

Hypoxia causes augmented formation of reactive oxygen species, which further causes lipid peroxidation [36, 41]. Lipid peroxidation creates various oxidative end-products, among which toxic aldehydes are the most dominant [18]. The major aldehyde product of lipid peroxidation is 4-HNE, believed to be the most detrimental aldehyde [18, 36], interacts with cellular macromolecules to produce a variety of protein adducts, leading to DNA damage, protein inactivation, and disease onset [18, 36]. ALDH2, an essential mitochondrial enzyme, is recognized for its crucial function in metabolism and protection against toxic agents, such as ROS and 4-HNE [42]. Studies have indicated that ALDH2 plays a protective role through the detoxification and clearance of 4-HNE in various oxidative stress-mediated cardiopulmonary diseases, such as myocardial ischemia/reperfusion, hypertension, and myocardial infarction [11, 12]. In the present study, we found remarkably augmented levels of 4-HNE in the lung tissue of ALDH2^−/−^ mice in response to hypoxia. This was accompanied by exacerbated pulmonary artery muscularization, right ventricular hypertrophy, fibrosis, and right-sided heart failure. Additionally, our *in vitro* studies also confirmed elevated 4-HNE levels in PASMCs after PDGF-BB treatment. These results suggest that 4-HNE is a detrimental element involved in the downstream signaling pathway related to the protective effects of ALDH2 in PH.

The pathological basis of hypoxia-induced PH involves pulmonary vasoconstriction and pulmonary vascular remodeling [25, 43, 44]. Abnormal PASMC migration and proliferation are key pathological features of pulmonary vascular remodeling due to persistent hypoxic PH. This pathological vascular remodeling is principally considered as medial thickening, increased muscularization, and luminal stenosis, all of which contribute to the progression of PH [19, 25]. Furthermore, previous studies have shown that factors regulating PASMC migration and proliferation protect against pathological medial thickening, vascular remodeling, and right ventricular pressure elevation [2, 45]. During the preparation of this manuscript, a study by Zhao et al. suggested that ALDH2 protects against hypoxia-induced PH by attenuating PASMC proliferation [18]. In this study, the wound healing, transwell, and EdU cell proliferation assays demonstrated that ALDH2 knockdown remarkedly augmented PASMC proliferation and migration. This was demonstrated by wound healing, transwell, and EdU cell proliferation assays. Additional immunoblot analysis further confirmed increased levels of PCNA and cyclin D1. Therefore, these results indicate that ALDH2 deficiency may promote right ventricular remodeling and failure by upregulating PASMC migration and proliferation.

Appropriate levels of autophagic activity are fundamental in maintaining cellular homeostasis through sequestration, turnover, and reprocessing of subcellular components including cytoplasmic substrates [46, 47]. Inappropriate autophagy results in the aggregation of toxic proteins and injured organelles. Conversely, extreme autophagy exceeding the necessity becomes destructive and results in cell death [46, 48]. Therefore, controversy remains on whether autophagy plays a beneficial or harmful role during PH. Lee et al. found increased expression of LC3B-II in the hypoxic mice lungs and the lungs of PH patients [24]. Consistently, several other studies have reported that the pharmacological inhibition of autophagy using drugs, such as NPS2390, puerarin, and apelin, suppresses PASMC proliferation [25, 49, 50]. Coherent to the previous studies, we demonstrated that the triggering of autophagy was involved in PASMC migration and proliferation. ALDH2 was reported to attenuate cardiovascular diseases through the regulation of autophagy including heart failure [16], diabetic cardiomyopathy [51], and myocardial dysfunction [52]. However, most studies emphasized on the direct detoxification properties of ALDH2 instead of its interactions with autophagy, especially in the scenario of PH. In our study, we found out for the first time that ALDH2 deficiency exacerbated autophagy as well as PASMC migration and proliferation, resulting in deteriorated ventricular function. Taken together, these findings suggest that ALDH2 protects against PH by inhibition of pathological PASMC migration and proliferation via the amelioration of aberrant autophagy.

The molecular mechanism of autophagy is complex and is regulated by various signaling pathways [46]. Particularly, the ERK1/2-Beclin-1 and PI3K-AKT-mTOR signaling pathways have been proven to regulate autophagy and the proliferation of PASMCs [53–55]. In this study, we found that both of these signaling pathways were stimulated. Furthermore, ALDH2 deficiency further exacerbated aberrant autophagic activity during the pathological process oh PH in lung tissues *in vivo* and in HPASMCs *in vitro* and enhanced the activation of these two signaling pathways. However, it is documented that the activation of ERK1/2-Beclin-1 pathway may promote autophagy whereas the activation of AKT-mTOR pathway is recognized to inhibit autophagy [26, 56]. Our negative findings of AKT-mTOR pathway in autophagy indicated an AKT-mTOR-independent mechanism in our current experimental settings. Consistently, it is implicated that AKT-mTOR (recognized as essential nutrients and energy indicator to regulate oxidative stress, protein synthesis, cell growth, and survival [57, 58]) has an essential role in autophagy-unrelated regulations of different physiological functions through activation of inflammatory responses and angiogenic processes [59]. Therefore, the proteinopathies of PH may be an inducer of AKT-mTOR pathway beyond autophagy regulation, or its influence was covered by enhanced ERK1/2-Beclin-1 dependent autophagy signaling pathway, similar to our previous study on AMPK in pressure overload injury [10].

Autophagy has been reported in previous studies to be associated with the activation of ERK-dependent signaling pathways in response to various stresses such as endoplasmic reticulum stress in lungs [60], amino acid reduction [61], autophagic vacuolation in tumors [62], aurintricarboxylic acid treatment in colon cancer cells [63], and cadmium-induced nephrotoxicity [64]. In addition, Beclin-1, a key regulator of autophagosome formation, serves as a platform protein that interacts with PI3K and plays an essential role in autophagy initiation and autophagic suppression of apoptosis [65, 66]. This characteristic is in line with the main feature of uncontrolled proliferation of PASMCs in pulmonary vascular remodeling of PH, evident in our result. A recent study by Xu et al. discovered that ALDH2 protects against oxidative stress by promoting autophagy also through the regulation of Beclin-1 in kidney injuries both *in vitro* and *in vivo*. Our results suggest a pivotal role of ERK1/2-Beclin-1-dependent regulation of autophagy in ALDH2-elicited inhibition of PASMC migration and proliferation. Nevertheless, further study is warranted to explore the precise mechanism of AKT-mTOR pathway in the ALDH2-induced regulation of PH and right-heart failure.

In conclusion, ALDH2 deficiency-induced autophagy is most possibly be mediated via the ERK1/2-Beclin-1 signaling pathway, suggesting it as a potential therapeutic target. A summary flow diagram showing the role and mechanisms of ALDH2 in the autophagy of PH is presented in Figure 6. Due to the lack of effective treatments for PH, this potential novel therapeutic target may be a new breakthrough.

Despite the impactful findings, there remains a limitation to our study. A possible medication to upregulate ALDH2 expression could be used to further verify the protective and therapeutic effects of PH. Further clinical studies are warranted to verify its applicability.

## 5. Conclusions

In summary, the stimulation of autophagy is involved in PASMC migration and proliferation and the pathological progression of PH. ALDH2 deficiency exacerbates this pathological progression in conjunction with increased ERK1/2 activity. Overall, our study suggests that ALDH2 could act as a unique therapeutic target for PH, probably via the regulation of autophagy and PASMC migration and proliferation.

## Figures and Tables

**Figure 1:** ALDH2 deficiency exacerbates PH in HySu mice. (a) RVSP in of normoxia (CON) and HySu-treated (PH) wild type (WT) and ALDH2^−/−^ (KO) mice. (b) Representative M-mode echocardiographic images of the morphology of right ventricles and RVEF statistical results of the four groups (WT CON, WT PH, KO CON, and KO PH). (c) Representative pulse wave echocardiographic images of pulmonary flow of the four groups (WT CON, WT PH, KO CON, and KO PH). (d) Pulmonary acceleration time of the four groups (WT CON, WT PH, KO CON, and KO PH). (e) The ratio of pulmonary acceleration time and pulmonary ejection time of the four groups (WT CON, WT PH, KO CON, and KO PH). Data are shown as mean ± SEM. ∗*p* < 0.05, ∗∗*p* < 0.01, ∗∗∗*p* < 0.001, ∗∗∗∗*p* < 0.0001, ns: not significant.

**Figure 2:** ALDH2 deficiency worsens the extent of PH and its effects on right ventricular remodeling and cardiomyocytes. (a) Gross morphology of hearts of normoxia (CON) and HySu-treated (PH) Wild type (WT) and ALDH2^−/−^ (KO) mice. (b) H&E longitudinal section staining of hearts and the quantification of the right ventricular hypertrophy index of the four groups (WT CON, WT PH, KO CON, and KO PH). (c) Electron microscopy examination of RV of the four groups (WT CON, WT PH, KO CON, and KO PH). (d) Representative images of RV by Masson collagen staining and the quantification of fibrosis of the four groups (WT CON, WT PH, KO CON, and KO PH). (e) Representative images of RV by WGA staining and the quantification of cross-sectional area of the four groups (WT CON, WT PH, KO CON, and KO PH). Data are shown as mean ± SEM. ∗*p* < 0.05, ∗∗*p* < 0.01, ∗∗∗*p* < 0.001, ∗∗∗∗*p* < 0.0001, ns: not significant.

**Figure 3:** ALDH2 deficiency exacerbates pulmonary vascular remodeling and oxidative damage in PH. (a) Representative images of H&E staining indicating the degree of muscularization (0–20% represents nonmuscularized, 20–40% partially muscularized, and 40–100% fully muscularized) of small pulmonary vessels from wild type (WT) and ALDH2^−/−^ (KO) mice treated with normoxia (CON) or HySu (PH). (b) Representative images of Masson staining indicating the area percentage of fibrosis area of mice lungs of the four groups (WT CON, WT PH, KO CON, and KO PH). (c) Western blot analysis of ALDH2, *α*SMA, and fibronectin of mice lungs of the four groups (WT CON, WT PH, KO CON, and KO PH). (d, e) Western blot analysis and quantification of (d) ALDH2 and (e) 4HNE of control (CON) and PDGF-BB- (PDGF-) treated vehicle (Lenti-NC) or ALDH2 knockdown (Lenti-ALDH2) HPASMCs. (f) Representative images of 4HNE immunohistochemical staining of mice lungs of the four groups (WT CON, WT PH, KO CON, and KO PH). Data are shown as mean ± SEM. ∗*p* < 0.05, ∗∗*p* < 0.01, ∗∗∗*p* < 0.001, ∗∗∗∗*p* < 0.0001, ns: not significant.

**Figure 4:** ALDH2 knockdown accentuates PASMC migration and proliferation in PH. (a) Representative photomicrographs of scratch assay and the quantification of the wound area of the control (CON) and PDGF-BB-treated (PDGF) vehicle (Lenti-NC) and ALDH2 knockdown (Lenti-ALDH2) HPASMCs. (b) Transwell experiment of the four groups of HPASMCs (Lenti-NC CON, Lenti-NC PDGF, Lenti-ALDH2 CON, and Lenti-ALDH2 PDGF) and their quantification results. (c) Western blot analysis of CyclinD1 and PCNA of the four groups of HPASMCs (Lenti-NC CON, Lenti-NC PDGF, Lenti-ALDH2 CON, and Lenti-ALDH2 PDGF) and quantification of the protein expression. (d) Representative fluorescence images and the quantification of EdU experiment of the four groups of HPASMCs (Lenti-NC CON, Lenti-NC PDGF, Lenti-ALDH2 CON, and Lenti-ALDH2 PDGF). Data are shown as mean ± SEM. ∗*p* < 0.05, ∗∗*p* < 0.01, ∗∗∗*p* < 0.001, ∗∗∗∗*p* < 0.0001, ns: not significant.

**Figure 5:** ALDH2 deficiency activates autophagy and its signaling pathways in PH. (a) Electron microscopy analysis of autophagic response in lung tissues of wild type (WT) and ALDH2^−/−^ (KO) mice treated with normoxia (CON) or HySu (PH). (Arrows indicate autophagosomes). (b) Representative images of LC3B immunohistochemical staining of lungs of the mice of WT CON, WT PH, KO CON, and KO PH groups. (c) Representative images of confocal fluorescence microscopy of the control (CON) or PDGF-BB-treated (PDGF) HPASMCs transfected with mRFP-GFP-LC3 adenovirus of the vehicle (Lenti-NC) and ALDH2 knockdown (Lenti-ALDH2) HPASMCs. (d) Western blot analysis of LC3B, P62, ATG5, ATG7, and Beclin1 and their quantification in the four HPASMCs groups (Lenti-NC CON, Lenti-NC PDGF, Lenti-ALDH2 CON, and Lenti-ALDH2 PDGF). (e) Western blot analysis of the phosphorylated state of PI3K, AKT, and mTOR and their quantification analyses in the four groups of HPASMCs (Lenti-NC CON, Lenti-NC PDGF, Lenti-ALDH2 CON, and Lenti-ALDH2 PDGF). (f) Western blot analysis of the phosphorylated state of ERK1/2 and its quantification analysis in the four groups of HPASMCs (Lenti-NC CON, Lenti-NC PDGF, Lenti-ALDH2 CON, and Lenti-ALDH2 PDGF). Data are shown as mean ± SEM. ∗*p* < 0.05, ∗∗*p* < 0.01, ∗∗∗p < 0.001, ∗∗∗∗p < 0.0001, ns: not significant.

**Figure 6:** Schematic of the mechanisms of ALDH2 protection against pulmonary hypertension.

## Data Availability

Data is available upon reasonable request from the corresponding author.

## References

[1] Humbert M., Sitbon O., Simonneau G. (2004). Treatment of pulmonary arterial hypertension. *The New England Journal of Medicine*.

[2] Tajsic T., Morrell N. W. (2010). Smooth muscle cell hypertrophy, proliferation, migration and apoptosis in pulmonary hypertension. *Comprehensive Physiology*.

[3] Liu X., Wang X., Pan Y. (2021). Artemisinin improves acetylcholine-induced vasodilatation in rats with primary hypertension. *Drug Design, Development and Therapy*.

[4] Sitbon O., Gomberg-Maitland M., Granton J. (2019). Clinical trial design and new therapies for pulmonary arterial hypertension. *The European Respiratory Journal*.

[5] Pan M., Han Y., Si R., Guo R., Desai A., Makino A. (2017). Hypoxia-induced pulmonary hypertension in type 2 diabetic mice. *Pulmonary circulation*.

[6] Nathan S. D., Barbera J. A., Gaine S. P. (2019). Pulmonary hypertension in chronic lung disease and hypoxia. *The European Respiratory Journal*.

[7] Guignabert C., Dorfmuller P. (2017). Pathology and pathobiology of pulmonary hypertension. *Seminars in Respiratory and Critical Care Medicine*.

[8] Zhang F., Chen A., Pan Y. (2022). Research progress on pulmonary arterial hypertension and the role of the angiotensin converting enzyme 2-angiotensin-(1-7)-mas axis in pulmonary arterial hypertension. *Cardiovascular Drugs and Therapy*.

[9] Shimoda L. A. (2020). Cellular pathways promoting pulmonary vascular remodeling by hypoxia. *Physiology (Bethesda)*.

[10] Shen C., Wang C., Fan F. (2015). Acetaldehyde dehydrogenase 2 (ALDH2) deficiency exacerbates pressure overload- induced cardiac dysfunction by inhibiting Beclin-1 dependent autophagy pathway. *Biochimica et Biophysica Acta*.

[11] Sun A., Cheng Y., Zhang Y. (2014). Aldehyde dehydrogenase 2 ameliorates doxorubicin-induced myocardial dysfunction through detoxification of 4-HNE and suppression of autophagy. *Journal of Molecular and Cellular Cardiology*.

[12] Chen C. H., Budas G. R., Churchill E. N., Disatnik M. H., Hurley T. D., Mochly-Rosen D. (2008). Activation of aldehyde dehydrogenase-2 reduces ischemic damage to the heart. *Science*.

[13] Sun A., Zou Y., Wang P. (2014). Mitochondrial aldehyde dehydrogenase 2 plays protective roles in heart failure after myocardial infarction via suppression of the cytosolic JNK/p53 pathway in mice. *Journal of the American Heart Association*.

[14] Sun X., Gao R., Li W. (2021). Alda-1 treatment promotes the therapeutic effect of mitochondrial transplantation for myocardial ischemia-reperfusion injury. *Bioactive materials*.

[15] Li X., Weng X., Shi H. (2019). Acetaldehyde dehydrogenase 2 deficiency exacerbates cardiac fibrosis by promoting mobilization and homing of bone marrow fibroblast progenitor cells. *Journal of Molecular and Cellular Cardiology*.

[16] Li W., Yin L., Sun X. (2020). Alpha-lipoic acid protects against pressure overload-induced heart failure via ALDH2-dependent Nrf1-FUNDC1 signaling. *Cell Death & Disease*.

[17] Zhang R., Wang J., Xue M., Xu F., Chen Y. (2017). ALDH2---the genetic polymorphism and enzymatic activity regulation: their epidemiologic and clinical implications. *Current Drug Targets*.

[18] Zhao Y., Wang B., Zhang J. (2019). ALDH2 (aldehyde dehydrogenase 2) protects against hypoxia-induced pulmonary hypertension. *Arteriosclerosis, Thrombosis, and Vascular Biology*.

[19] Xu T., Liu S., Ma T., Jia Z., Zhang Z., Wang A. (2017). Aldehyde dehydrogenase 2 protects against oxidative stress associated with pulmonary arterial hypertension. *Redox Biology*.

[20] Mizushima N., Komatsu M. (2011). Autophagy: renovation of cells and tissues. *Cell*.

[21] Nishida K., Otsu K. (2016). Autophagy during cardiac remodeling. *Journal of Molecular and Cellular Cardiology*.

[22] Kamareddine L., Ghantous C. M., Allouch S. (2021). Between inflammation and autophagy: the role of leptin-adiponectin axis in cardiac remodeling. *Journal of Inflammation Research*.

[23] Miyamoto S. (2019). Autophagy and cardiac aging. *Cell Death and Differentiation*.

[24] Lee S. J., Smith A., Guo L. (2011). Autophagic protein LC3B confers resistance against hypoxia-induced pulmonary hypertension. *American Journal of Respiratory and Critical Care Medicine*.

[25] Peng X., Wei C., Li H. Z. (2019). NPS2390, a selective calcium-sensing receptor antagonist controls the phenotypic modulation of hypoxic human pulmonary arterial smooth muscle cells by regulating autophagy. *Journal of Translational Internal Medicine*.

[26] Gu J., Hu W., Song Z. P., Chen Y. G., Zhang D. D., Wang C. Q. (2016). Rapamycin inhibits cardiac hypertrophy by promoting autophagy via the MEK/ERK/Beclin-1 pathway. *Frontiers in Physiology*.

[27] Kitagawa K., Kawamoto T., Kunugita N. (2000). Aldehyde dehydrogenase (ALDH) 2 associates with oxidation of methoxyacetaldehyde; in vitro analysis with liver subcellular fraction derived from human and Aldh2 gene targeting mouse. *FEBS Letters*.

[28] Liu X., Sun X., Liao H. (2015). Mitochondrial aldehyde dehydrogenase 2 regulates revascularization in chronic ischemia: potential impact on the development of coronary collateral circulation. *Arteriosclerosis, Thrombosis, and Vascular Biology*.

[29] Perros F., Montani D., Dorfmuller P. (2008). Platelet-derived growth factor expression and function in idiopathic pulmonary arterial hypertension. *American Journal of Respiratory and Critical Care Medicine*.

[30] Schermuly R. T., Dony E., Ghofrani H. A. (2005). Reversal of experimental pulmonary hypertension by PDGF inhibition. *The Journal of Clinical Investigation*.

[31] Barst R. J. (2005). PDGF signaling in pulmonary arterial hypertension. *The Journal of Clinical Investigation*.

[32] Sweatt A. J., Hedlin H. K., Balasubramanian V. (2019). Discovery of distinct immune phenotypes using machine learning in pulmonary arterial hypertension. *Circulation Research*.

[33] Ntokou A., Dave J. M., Kauffman A. C. (2021). Macrophage-derived PDGF-B induces muscularization in murine and human pulmonary *hypertension*. *Insight*.

[34] Yu T., Guo F., Yu Y. (2017). *Fusobacterium nucleatum* promotes chemoresistance to colorectal cancer by modulating autophagy. *Cell*.

[35] Wang K. K., Posner A., Hajimohammadreza I. (1996). Total protein extraction from cultured cells for use in electrophoresis and western blotting. *BioTechniques*.

[36] Ayala A., Munoz M. F., Arguelles S. (2014). Lipid peroxidation: production, metabolism, and signaling mechanisms of malondialdehyde and 4-hydroxy-2-nonenal. *Oxidative Medicine and Cellular Longevity*.

[37] Ryter S. W., Nakahira K., Haspel J. A., Choi A. M. (2012). Autophagy in pulmonary diseases. *Annual Review of Physiology*.

[38] Ichimiya T., Yamakawa T., Hirano T. (2020). Autophagy and autophagy-related diseases: a review. *International Journal of Molecular Sciences*.

[39] Klionsky D. J., Petroni G., Amaravadi R. K. (2021). Autophagy in major human diseases. *The EMBO Journal*.

[40] Chen C. H., Ferreira J. C. B., Mochly-Rosen D. (2019). ALDH2 and cardiovascular disease. *Advances in Experimental Medicine and Biology*.

[41] Su L. J., Zhang J. H., Gomez H. (2019). Reactive oxygen species-induced lipid peroxidation in apoptosis, autophagy, and ferroptosis. *Oxidative Medicine and Cellular Longevity*.

[42] Hink U., Daiber A., Kayhan N. (2007). Oxidative inhibition of the mitochondrial aldehyde dehydrogenase promotes nitroglycerin tolerance in human blood vessels. *Journal of the American College of Cardiology*.

[43] Pan Y., Sun S., Wang X. (2021). Improvement of vascular function by knockdown of salusin-*β* in hypertensive rats via nitric oxide and reactive oxygen species signaling pathway. *Frontiers in Physiology*.

[44] Zhang F., Xu Y., Pan Y. (2019). Effects of angiotensin-(1-7) and angiotensin II on acetylcholine-induced vascular relaxation in spontaneously hypertensive rats. *Oxidative Medicine and Cellular Longevity*.

[45] Huetsch J. C., Suresh K., Shimoda L. A. (2019). Regulation of smooth muscle cell proliferation by NADPH oxidases in pulmonary hypertension. *Antioxidants*.

[46] Nakahira K., Pabon Porras M. A., Choi A. M. (2016). Autophagy in pulmonary diseases. *American Journal of Respiratory and Critical Care Medicine*.

[47] Zhou Y., Wang Y., Wang X. (2017). The protective effects of kappa-opioid receptor stimulation in hypoxic pulmonary hypertension involve inhibition of autophagy through the AMPK-MTOR pathway. *Cellular Physiology and Biochemistry*.

[48] Lavandero S., Chiong M., Rothermel B. A., Hill J. A. (2015). Autophagy in cardiovascular biology. *The Journal of Clinical Investigation*.

[49] Zhang X. D., Wang L. W., Wang S. J. (2015). Effect of puerarin on hypoxia induced proliferation of PASMCs by regulating reactive oxygen. *Zhongguo Zhong Yao Za Zhi*.

[50] Zhang H., Gong Y., Wang Z. (2014). Apelin inhibits the proliferation and migration of rat PASMCs via the activation of PI3K/Akt/mTOR signal and the inhibition of autophagy under hypoxia. *Journal of Cellular and Molecular Medicine*.

[51] Lee H. L., Hee S. W., Hsuan C. F. (2021). A novel ALDH2 activator AD-9308 improves diastolic and systolic myocardial functions in streptozotocin-induced diabetic mice. *Antioxidants*.

[52] Ji W., Wan T., Zhang F., Zhu X., Guo S., Mei X. (2021). Aldehyde dehydrogenase 2 protects against lipopolysaccharide-induced myocardial injury by suppressing mitophagy. *Frontiers in Pharmacology*.

[53] Shi Y., Gu C., Zhao T. (2021). Combination therapy with rapamycin and low dose imatinib in pulmonary hypertension. *Frontiers in Pharmacology*.

[54] Gredic M., Wu C. Y., Hadzic S. (2022). Myeloid cell-specific deletion of inducible nitric oxide synthase protects against smoke-induced pulmonary hypertension in mice. *The European Respiratory Journal*.

[55] Su Y., Han W., Kovacs-Kasa A., Verin A. D., Kovacs L. (2021). HDAC6 activates ERK in airway and pulmonary vascular remodeling of chronic obstructive pulmonary disease. *American Journal of Respiratory Cell and Molecular Biology*.

[56] Ma H., Guo R., Yu L., Zhang Y., Ren J. (2011). Aldehyde dehydrogenase 2 (ALDH2) rescues myocardial ischaemia/reperfusion injury: role of autophagy paradox and toxic aldehyde. *European Heart Journal*.

[57] Li Q., Ren J. (2006). Cardiac overexpression of metallothionein rescues chronic alcohol intake-induced cardiomyocyte dysfunction: role of Akt, mammalian target of rapamycin and ribosomal p70s6 kinase. *Alcohol and Alcoholism*.

[58] Ma J., Meng Y., Kwiatkowski D. J. (2010). Mammalian target of rapamycin regulates murine and human cell differentiation through STAT3/p63/Jagged/Notch cascade. *The Journal of Clinical Investigation*.

[59] Ghafouri-Fard S., Khanbabapour Sasi A., Hussen B. M. (2022). Interplay between PI3K/AKT pathway and heart disorders. *Molecular Biology Reports*.

[60] Oh S. H., Lim S. C. (2009). Endoplasmic reticulum stress-mediated autophagy/apoptosis induced by capsaicin (8-methyl-N-vanillyl-6-nonenamide) and dihydrocapsaicin is regulated by the extent of c-Jun NH2-terminal kinase/extracellular signal-regulated kinase activation in WI38 lung epithelial fibroblast cells. *The Journal of Pharmacology and Experimental Therapeutics*.

[61] Ogier-Denis E., Pattingre S., El Benna J., Codogno P. (2000). Erk1/2-dependent phosphorylation of G*α*-interacting protein stimulates its GTPase accelerating activity and autophagy in human colon cancer cells∗. *The Journal of Biological Chemistry*.

[62] Corcelle E., Nebout M., Bekri S. (2006). Disruption of autophagy at the maturation step by the carcinogen lindane is associated with the sustained mitogen-activated protein kinase/extracellular signal-regulated kinase activity. *Cancer Research*.

[63] Pattingre S., Bauvy C., Codogno P. (2003). Amino acids interfere with the ERK1/2-dependent control of macroautophagy by controlling the activation of Raf-1 in human colon cancer HT-29 cells∗. *The Journal of Biological Chemistry*.

[64] Yang L. Y., Wu K. H., Chiu W. T., Wang S. H., Shih C. M. (2009). The cadmium-induced death of mesangial cells results in nephrotoxicity. *Autophagy*.

[65] Jiang S., Guo R., Zhang Y., Zou Y., Ren J. (2013). Heavy metal scavenger metallothionein mitigates deep hypothermia-induced myocardial contractile anomalies: role of autophagy. *American Journal of Physiology. Endocrinology and Metabolism*.

[66] Maejima Y., Kyoi S., Zhai P. (2013). Mst1 inhibits autophagy by promoting the interaction between Beclin1 and Bcl-2. *Nature Medicine*.

